# Efficacy of Applying Kanglaite Injection under Incentive Nursing Intervention in Treating Patients with Advanced Penile Carcinoma and Its Effect on Treatment Compliance

**DOI:** 10.1155/2021/4114658

**Published:** 2021-10-25

**Authors:** Juan Wang, Qingyan Liu, Mei Hong, Ge Li, Yong Cheng

**Affiliations:** ^1^Department of Operating Room, Affiliated Hospital of Southwest Medical University, Luzhou, Sichuan, China; ^2^Department of Urology Surgery, Affiliated Hospital of Southwest Medical University, Luzhou, Sichuan, China

## Abstract

**Objective:**

To explore the efficacy of applying Kanglaite (KLT) injection under incentive nursing intervention (INI) in treating patients with advanced penile carcinoma and its effect on patient treatment compliance.

**Methods:**

The clinical data of 120 patients with advanced penile carcinoma treated in the Affiliated Hospital of Southwest Medical University from February 2019 to February 2020 were retrospectively analyzed, and the patients were equally divided into the experimental group (*n* = 60) and control group (*n* = 60) according to their admission order. All patients received the KLT injection treatment; those in the control group accepted the conventional nursing; and on this basis, those in the experimental group accepted INI, including psychological nursing intervention, which was conducted concurrently with the treatment, to compare their short-term efficacy, treatment compliance, degree of cancer-related fatigue (Brief Fatigue Inventory), and negative emotion scores (Hospital Anxiety and Depression Scale) between the two groups.

**Results:**

Compared with the control group, the experimental group presented a significantly higher objective remission rate (58.3%) (*P* < 0.05), higher rates of excellent and good treatment compliance (*P* < 0.05), and lower degree of cancer-related fatigue and negative emotion scores (*P* < 0.001).

**Conclusion:**

INI can improve the negative emotions in patients with advanced carcinoma of the penis, alleviate their degree of cancer-related fatigue, promote their treatment compliance, and achieve a more significant efficacy of applying the KLT injection treatment, so it should be promoted in practice.

## 1. Introduction

Carcinoma of the penis is a malignant tumor that originates from the glans penis, coronal sulcus, the mucosa of the prepuce inner plate, and the skin of the penis, with an incidence accounting for more than 90% of all penile tumors [1, 2]. At present, academia has not clarified the pathogenic factor, but it is believed that smegma, chronic inflammatory stimulation, and so on are closely related to its incidence [3, 4]. In general, early penile cancer is less malignant, and patients can achieve a surgical cure rate of 75% [5]. However, advanced penile cancer patients with inguinal lymph node metastasis only have a 5-year survival rate of 20%, and may even die within 2 years in case of no comprehensive therapeutic measures [6, 7]. Therefore, additional therapeutic measures should be performed for such patients based on chemotherapy. Kanglaite (KLT) injection is a common drug used in the clinic for treating malignant tumors, which mainly contains coix seed oil, granulesten, and glycerol for injection, of which coix seed is a bidirectional broad-spectrum anticancer injection emulsion that can effectively enhance the patients' immune function and at the same time inhibit the proliferation of malignant tumor cells [8]. Clinical studies have shown that KLT injection can improve the quality of life and increase the short-term survival rate of patients, but it has no obvious improvement on the psychological condition of patients [9].

Affected by social culture, medical conditions, family conditions, and other subjective and objective factors, patients with advanced penile cancer usually face great physical and mental stress, and long-term psychological stress will lead to neurological disorders in patients, which will eventually trigger somatic symptoms and result in decreased treatment effect. To improve the psychological status of patients, some scholars have proposed the incentive nursing intervention (INI) in practice [10], which refers to effective education, guidance, and emotional support for the specific physical and mental conditions of patients and high-quality nursing personnel, thereby helping patients with building confidence and improving treatment compliance [11]. No studies on the application of INI in treating advanced penile cancer patients with KLT injection have been conducted in previous literature. Based on this, the efficacy of adopting KLT injection treatment under INI in treating such patients and its effect on patient treatment compliance were explored herein, with the results reported below.

## 2. Data and Methods

### 2.1. Study Design

It was a retrospective study and conducted from February 2019 to February 2020 in Affiliated Hospital of Southwest Medical University to explore the efficacy of adopting KLT injection treatment under INI in treating patients with advanced carcinoma of the penis and its effect on patient treatment compliance.

### 2.2. Enrolment of Research Objects

The clinical data of patients with advanced carcinoma of the penis treated in Affiliated Hospital of Southwest Medical University from February 2019 to February 2020 were retrospectively analyzed. The patients were included according to the following criteria: (1) the patients were diagnosed with penile carcinoma after biopsy [12] and were in stage III or IV according to the Jackson staging method [13]; (2) the patients were treated in our hospital throughout, with no occurrence of death, transfer, and discontinuation of therapy; (3) the patients had complete clinical data; and (4) the patients did not have other serious complications. The patients were excluded according to the following criteria: (1) the patients were unable to communicate with others because of hearing disorder, language disorder, unconsciousness, or mental diseases; (2) during treatment, the patients quit, died, changed the treatment regimen, or were found missing in the follow-up visit; (3) the patients suffered from other serious organic diseases; and (4) the patients' clinical data were incomplete.

### 2.3. Steps

A total of 120 patients were included in the study and equally divided into the experimental group and control group according to their admission order, with 60 cases each. On the day that the patients agreed to join the study, the study team collected their sociodemographic data and clinical performance data, and the nursing personnel made no implications except for explaining the questionnaires; after filling, the questionnaires were taken back and verified for completeness, and such process was repeated after the end of nursing. In case of any omissions, the patients were encouraged to complete the questionnaires based on no violation of the voluntary principle to ensure integrity and authenticity.

### 2.4. Moral Consideration

The study met the principle of the World Medical Association Declaration of Helsinki [12] and was approved by the ethics committee of Affiliated Hospital of Southwest Medical University. The study team explained the purpose, meaning, content, and confidentiality of the study to the enrolled patients, and the patients signed the informed consent.

### 2.5. Criteria of Quitting the Experiment

For the patients with one of the following situations and who were judged unsuitable for continuously accepting the experiment by the study team, their case records would be reserved but not used for data analysis: (1) those who experienced adverse events or serious adverse events; (2) those who presented condition worsened during the experiment; (3) subjects developed certain severe comorbidities or complications; and (4) subjects were unwilling to continue with the clinical trial and proposed the request of withdrawal from the clinical trial to the study team.

### 2.6. Methods

All patients received two courses of KLT injection treatment; that is, 200 ml of KLT injection (manufactured: Zhejiang Kanglaite Pharmaceutical Co., Ltd.; NMPA approval no. Z10970091) was administered once daily via slow intravenous infusion for 21 d as one course, and the next course was proceeded 5 days after the end of the first course.

Meanwhile, the patients in the control group received conventional nursing; namely, their vital signs were closely monitored and guidance for diet, exercise, drug use, and so on was given, with the specific methods. (1) Drug use: the patients with carcinoma of the penis usually felt pain at the penis and scrotum, so the nursing personnel could administer the paracetamol oxycodone sustained-release tablets (manufactured: China National Pharmaceutical Industry Corporation Ltd.; NMPA approval no: J20171086) to the patients under medical supervision and at the same time perform continuous infusion with a micro analgesic pump, establish the nursing record on observation of micro analgesic pump and multipurpose administration to effectively monitor the patients' condition, and pay special attention to the adverse reactions after administration, and for patients with local swelling, their infusion part should be changed in time. According to the medical advice, the nursing personnel needed to help the patients with perineal tumor rupture in changing their dressings twice a day in strict accordance with the aseptic operation; the dressings were fully soaked with 0.9% normal saline before changing to avoid pain sensation and bleeding, the thickness of sterile gauze for cover should be appropriate to avoid infection, and the frequency of dressing changing could be increased if necessary based on the dressing status. The dressing condition at the tumor was observed regularly after dressing change, and the corresponding records were made. (2) Preventing adverse reactions: for patients with constipation, the nursing personnel could give them laxatives and glycerine enema (if necessary), help them with forming a normal bowl evacuation habit, repeatedly advise them to eat more food with crude fiber, fresh fruits, and vegetables, and increase exercise frequency, and in case of diarrhea, the patients should inform the nursing personnel immediately. For patients with edema of both lower limbs, the nursing personnel should give them diuretic drugs, help them with massage and turning over, and repeatedly advise them to avoid sitting for a long time to prevent skin rupture. For patients with vomiting, the nursing personnel should give them drugs that inhibit gastric acid, ask the family members of the patients to prepare light food, and inform the patients of avoiding hypertense. (3) Health education: the nursing personnel distributed the health education handbooks prepared by our hospital to the patients and popularized the relevant knowledge about carcinoma of the penis to the patients and their family members to improve their self-care ability and alleviate their negative emotions.

On this basis, INI was implemented to the patients in the experimental group with the following methods: (1) the nursing personnel were trained by a professional psychologist to comprehensively learn to help the patients with alleviating their negative emotions by incentive methods such as making use of target, emotion, and materials and to promote the scientific nature and professionalism of INI with evidence-based nursing. (2) After admission, the one-on-one mental intervention by nursing personnel was conducted on the patients in the experimental group. The nursing personnel first carefully read the patients' basic information and then prepared corresponding nursing plans according to the patients' condition, educational degree, personality, and mental state, to provide them with specific health education and emotional support with individual differences. (3) The patients with advanced carcinoma of the penis were prone to negative emotions such as dysesthesia and anxiety, so the nursing personnel should pay attention to the changes in their mental state and emotions, increase the frequency of communicating with them, and explain relevant knowledge about the disease in one-on-one communication, thereby relieving their negative emotions and promoting their treatment compliance. (4) Before chemotherapy, the nursing personnel should carefully listen to the patients' demands, encourage them through verbal communication, and help them with solving their reasonable demands, to reduce their anxiety and enable them to build confidence; after solving the problems, praises and encouragement were given to the patients, so that they could bravely share their problems, fully understand their value, face the difficulties and challenges brought by treatment in a more positive way, and reduce their worries. (5) The nursing personnel set phased targets and good examples for the patients and praised the patients when they finished every small target and made any progress. (6) The nursing personnel needed to think about the patients, keep a sincere and caring attitude, and feel for the patients during communication, thus enabling the patients to promote their trust in the nursing personnel and then increase treatment compliance.

### 2.7. Observation Criteria

#### 2.7.1. General Information

The general information extraction forms were created by the patients themselves, including the in-patient number, name, age, body mass, BMI, cancer stage, method of paying medical fees, marital status, monthly income, educational degree, place of residence, and living habits.

#### 2.7.2. Short-Term Efficacy

According to the Response Evaluation Criteria in Solid Tumors (RECICT) established by WHO in 2000 [14], the patients' condition was classified into complete response (CR, disappearance of lesions, no new lesions, and tumor markers restored to normal for over one month), partial response (PR, ≥30% decrease in SLD (the sum of the longest diameters of target lesion) for over one month), stable disease (SD, no PR-no PD), and progressive disease (PD, ≥20% increase in SLD, or new lesions). The treatment effect of patients was compared by the objective remission rate (ORR, CR + PR) and disease control rate (DCR, CR + PR + SD).

#### 2.7.3. Treatment Compliance

It was considered as excellent compliance in case that the patients fully accepted the treatment regimen established by the physician and the nursing regimen established by the nursing personnel, went through the treatment smoothly, and cooperated with various nursing measures; good compliance in case that the patients basically accepted the treatment regimen established by the physician and the nursing regimen established by the nursing personnel, finished the most of the treatment and cooperated with various nursing measures from time to time; and poor compliance in case that the patients only cooperated with the treatment when the disease was aggravated or, once in a while, could not understand various adverse reactions occurred during treatment and failed to cooperate with the nursing measures. After nursing, the treatment compliance of patients in both groups was compared.

#### 2.7.4. Degree of Cancer-Related Fatigue

The degree of cancer-related fatigue of patients before and after treatment was evaluated by the Brief Fatigue Inventory (BFI) [15], which has been validated in international literature for its credibility and sensitivity. On a scale of 0–10 points, 0 points indicated no fatigue, 1–3 points indicated mild fatigue, 4–6 points indicated medium fatigue, and 7–10 points indicated severe fatigue.

#### 2.7.5. Negative Emotion Scores

The emotional state of patients before and after treatment was evaluated by Hospital Anxiety and Depression Scale (HAD) [16], which has been validated in international literature for its credibility and sensitivity. On a scale of 0–42 points, 0 points indicated no anxiety, and higher scores indicated the more serious anxiety and depression.

### 2.8. Statistical Processing

In this study, the data processing software was SPSS20.0, the picture drawing software was GraphPad Prism 7 (GraphPad Software, San Diego, USA), items included were enumeration data and measurement data, methods used were *X*^2^ test and *t*-test, and differences were considered statistically significant at *P* < 0.05.

## 3. Results

### 3.1. Comparison of Patients' General Information

No statistical differences in the patients' general information between the two groups were observed (*P* > 0.05). See Table 1.

### 3.2. Comparison of Patients' Short-Term Efficacy

The ORR of the experimental group was 58.3%, which was remarkably higher than that of the control group (*P* < 0.05). See Table 2.

### 3.3. Comparison of Patients' Treatment Compliance

The rates of excellent and good treatment compliance of patients were higher in the experimental group than in the control group (*P* < 0.05). See Figure 1.

The numbers of patients with excellent, good, and poor treatment compliance in the experimental group were 48 (80.0%), 10 (16.7%), and 2 (3.3%), respectively; and the numbers of patients with excellent, good, and poor treatment compliance in the control group were 35 (58.3%), 13 (21.7%), and 12 (20.0%), respectively.

### 3.4. Comparison of Patients' Degree of Cancer-Related Fatigue and Negative Emotion Scores

Compared with the control group after treatment, the patients' degree of cancer-related fatigue and negative emotion scores of the experimental group were significantly lower (*P* < 0.001). See Figure 2.

Figure 2(a) shows the BFI scores. The horizontal axis from left to right denotes before and after nursing; the lines with dots indicated the experimental group, and the lines with blocks indicated the control group. Before nursing, the BFI scores between the two groups were not statistically different (7.21 ± 1.23 vs. 7.23 ± 1.20, *P* > 0.05); and after nursing, the BFI scores were significantly lower in the experimental group than in the control group (5.10 ± 0.54 vs. 6.15 ± 0.65, *P* < 0.001).

Figure 2(b) shows the HAD scores. The horizontal axis from left to right denotes before and after nursing; the lines with dots indicated the experimental group, and the lines with blocks indicated the control group. Before nursing, the HAD scores between the two groups were not statistically different (34.65 ± 2.21 vs. 34.68 ± 2.23, *P* > 0.05); and after nursing, the HAD scores were significantly lower in the experimental group than in the control group (19.65 ± 1.68 vs. 26.98 ± 2.54, *P* < 0.001).

## 4. Discussion

Penile cancer is the most common malignant neoplasm of the penis. At present, academia has not clarified the pathogenic factor of penile cancer, but it is generally assumed that phimosis, redundant prepuce, smegma, chronic inflammation, and so on are closely related, and country and region, ethnic folklore, religion, and life habits also affect the incidence to a certain extent [17]. In the 1950s, the incidence of penile cancer in China ranked first in the male reproductive system malignancies, while, with increasing medical and health technologies nowadays, penile cancer has become a rare male tumor, with an incidence that accounts for only 1.0% of all male malignancies [18]. Clinical practice shows that most penile cancers are less malignant, and the cure rate can reach up to 80.0% in patients at the early stage of the disease, but advanced penile cancer patients with distant metastasis have a 5-year survival rate of only 20% [19] and poor prognosis. Chemotherapy is the main treatment modality for patients with advanced penile cancer because it can prolong the survival time of the patients, but it usually triggers organic responses in patients and leads to more serious psychological stress. Compared with conventional chemotherapeutic agents including pingyangmycin and 5-fluorouracil, KLT injection is safer and can accelerate the apoptosis of malignant cells, reduce the frequency of mitosis, and be beneficial in improving the comprehensive efficacy based on chemotherapy. However, advanced penile cancer usually causes severe mental irritation to patients, who will not only feel anxious and tense due to the medical economic burden, but also develop negative and hostile feelings caused by the ulcerated and malodorous penis, and some patients will even experience somatic symptoms due to the long-term poor mental health, leading to further reduced treatment adherence that is not conducive to the performance of clinical treatment and nursing.

As the concept of medical treatment has been changed in Chinese residents, the psychological state of patients with advanced cancer has become a recognized evaluation criterion for efficacy in the academic community [20], the nursing model solely centered on treatment can no longer meet the needs of clinical care, and the more targeted nursing based on humanities care and with remodeling of the patients' personality and dignity as an essence has become the important development direction in the care of such patients. INI is the more common nursing model for cancer patients in recent years, which aims to integrate emotional and physical support into all aspects of nursing, to make patients fully feel the care of nursing personnel, and thus be more cooperative with the nursing personnel's actions during clinical treatment [21]. The study by scholars Patel et al. showed that performing INI for patients with malignant tumors could reduce their scores of Anxiety Self-Rating Scale and Depression Self-Rating Scale [22], and this study also found that patients in the experimental group had a significantly lower degree of cancer-related fatigue and negative emotion scores after nursing than those in the control group (*P* < 0.001), indicating that the nursing model was people-centered, practically felt for the patients, and stimulated the patients' positive mental state, thereby keeping their body in a highly excited state, enhancing their confidence in conquering the disease, and relieving their negative emotions. In many references, it was shown that negative emotions were important factors affecting patient treatment compliance, which was the key to ensuring the implementation of medical behaviors and nursing measures, and poor compliance could result in tumor recurrence and metastasis and seriously affect patient prognosis [23]. With INI, the penile cancer-related knowledge could be popularized through one-to-one communication for patients to form a more clear perception of the condition, which was beneficial for enhancing the clinical management efficacy of the nursing personnel, and therefore the rates of excellent and good treatment compliance were significantly higher in the experimental group than in the control group (*P* < 0.05). The studies by scholars Mehta et al. showed that a good nurse-patient relationship was the basis of treatment [24], and INI could enhance patients' trust in nursing personnel, maintain their correct expectations during treatment, and promote their cooperation, so the ORR of the experimental group was significantly higher than that of the control group (*P* < 0.05), denoting INI could sufficiently mobilize patients' enthusiasm and reduce the adverse effects of their negative emotions and hostility to the treatment, thus achieving better therapeutic outcomes.

## 5. Conclusion

Based on KLT injection treatment, INI can ease the negative emotions in patients with advanced carcinoma of the penis, improve their degree of cancer-related fatigue, promote their treatment compliance, and achieve a more desirable treatment effect so such nursing method should be promoted in practice.

## Figures and Tables

**Figure 1:** Comparison of patients' treatment compliance (*n*(%)). The black areas indicated excellent treatment compliance, the light gray areas indicated good treatment compliance, and the dark gray areas indicated poor treatment compliance. (a) Experimental group and (b) control group.

**Figure 2:** Comparison of patients' degree of cancer-related fatigue and negative emotion scores ($\bar{x}\pm s$, points). # means *P* < 0.001.

**Table 1:** Comparison of patients' general information.

Group	Experimental (*n* = 60)	Control (*n* = 60)	*X* ^2^/*t*	*P*
Age (years)				
Range	35–74	34–76		
Mean age	60.12 ± 3.65	59.87 ± 3.54	0.381	0.704
Mean body weight (kg)	59.56 ± 2.54	59.17 ± 2.57	0.836	0.405
BMI (kg/m^2^)	23.98 ± 1.65	23.88 ± 1.58	0.339	0.735
Cancer stage			0.139	0.709
III	35	37		
IV	25	23		
Payment method for medical fee				
Medical insurance	32	30	0.134	0.715
Commercial insurance	20	18	0.154	0.695
Others	8	12	0.960	0.327
Marital status			0.196	0.658
Married	46	48		
Unmarried/divorced/widowed	14	12		
Place of residence			0.034	0.855
Urban area	28	27		
Rural area	32	33		
Monthly income (yuan)			0.035	0.853
≥4000	25	24		
<4000	35	36		
Life habit				
Smoking history	30	28	0.134	0.715
Drinking history	27	29	0.134	0.714
Educational degree			0.034	0.854
Senior high school and below	26	27		
College and above	34	33		

**Table 2:** Comparison of patients' short-term efficacy (*n* (%)).

Group	CR	PR	SD	PD	ORR	DCR
Experimental	5 (8.3)	30 (50.0)	15 (25.0)	10 (16.7)	35 (58.3)	50 (83.3)
Control	0 (0.0)	24 (40.0)	18 (30.0)	18 (30.0)	24 (40.0)	42 (70.0)
*X* ^2^	5.217	1.212	0.376	2.981	4.034	2.981
*P*	0.022	0.271	0.540	0.084	0.045	0.084

## Data Availability

The data used to support the findings of this study are available on reasonable request from the corresponding author.
